The article "Effect of Palonosetron on Physical Symptoms of Surgical Patients: A Systematic Review and Meta-Analysis" was published in 2022. Journal: Comput Math Methods Med.

# Effect of Palonosetron on Physical Symptoms of Surgical Patients: A Systematic Review and Meta-Analysis

**DOI:** 10.1155/2022/7474053

**Published:** 2022-03-27

**Authors:** Ruichao Chu

**Affiliations:** Shandong Maternal and Child Health Hospital Anesthesiology Department, 250000 Jinan, China

## Abstract

**Background:**

Postoperative nausea and vomiting (PONV) is a typical and unpleasant physical symptom that occurs in patients after surgery, and it may be one of the most challenging elements of the recovery process. PONV can be caused by a variety of factors, including surgery itself, anesthesia, or medications. Palonosetron is a medication that is now licensed by the Food and Drug Administration for the treatment of this ailment. The efficacy of palonosetron in reducing physical symptoms in patients following surgery was investigated in this meta-analysis and comprehensive review.

**Methods:**

Following a quick search of databases such as CENTRAL, EMBASE, CINAHL, Google Scholar, the Science quotation index's Web site, the United States clinical trial check-in, the United Kingdom clinical trial check-in, the New Zealand clinical trial check-in, and the Australia check-in, as well as outlines of major anesthesia meetings held in the previous five years, we were able to get a good start on our research. Growing adults who had surgery and were given other drugs were compared to individuals who did get palonosetron in randomized controlled trials.

**Results:**

A total of 8324 participants were recruited in 10 different clinical studies. It has been shown that palonosetron may significantly reduce the 24-hour PONV incidence and 95% confidence interval (CI) 0.41–0.86. When comparing the 6-hour and 48-hour time periods, the incidences of experiencing PONV were neither statistically different (RR: 0.82, 95% confidence interval: 0.61–1.09) or considerably different (RR: 0.60, 95% confidence interval: 0.33–1.10). Following in a similar vein, there was no significant difference between the groups in the occurrence of PONV after 48 hours (RR: 0.82, 95 percent CI: 0.59–1.14). The most often reported side effects of the medicine were headaches and dizziness, which were the most common. Regardless of the drug used, the difference in adverse reactions was not statistically significant.

**Conclusion:**

When it comes to the prevention of early PONV, it has been shown that palonosetron is more effective than other medications. Palonosetron, on the other hand, has been demonstrated to be more effective than other medications in preventing vomiting after laparoscopic surgery.

## 1. Introduction

A large rise in the number of patients who successfully complete surgery has resulted from the introduction of more powerful medications into anesthesia in recent decades [1]. As many as 70 percent of surgical patients have vomiting or postoperative nausea and vomiting (PONV), which are two of the most common anesthetic difficulties [2], after surgery. There have been reports of PONV being associated with the activation of four vomiting centers, including the vestibular system, the chemoreceptor trigger area, the gastro-intestinal vagal fear system, and the cortical plaza. The vestibular system is composed of four components [3]. A multitude of neurotransmitters are responsible for transmitting nerve impulses and information from these four zones to the vomiting mall in the medulla. A cascade of somatic and visceral reactions, including nausea and vomiting, occurs whenever a section of the body is harmed [4, 5]. Acute esophageal rips and hernias, pneumonia, and pneumothorax are among the complications associated with PONV exposure. Aside from these side effects, PONV may also cause dehydration and anxiety, as well as acid-base imbalance and electrolyte imbalance. This means that PONV in surgical patients must be avoided at all costs [5]. Preventing PONV following surgery may help patients stay hydrated after surgery while also minimizing the demand on hospital resources and infrastructure. In recent research, it has been shown that antiemetic 5-HT3 antagonists may be beneficial in the prevention of postoperative nausea and vomiting (PONV) [6]. As a result, these drugs are now routinely used to prevent PONV in a variety of conditions [7]. Among the most often prescribed drugs in today's medical world are the 5-HT3 receptor antagonist pharmaceuticals ondansetron, ramosetron, tropisetron, and granisetron. As a new 5-HT3 receptor antagonist with a long half-life, palonosetron hydrochloride has the potential to be used as a prospective treatment [8]. The use of palonosetron for the prevention of PONV was authorized by the United States Food and Drug Administration in 2003. After it was approved for usage, palonosetron became extensively utilized in clinical practice across the globe almost immediately. Compared to other medications, palonosetron has a much longer half-life (about 40 hours) and has a significantly greater affinity for the 5-HT3 receptor, with an affinity that ranges from a factor of 30 to 100 [9]. A recent study on the usefulness of palonosetron in avoiding postoperative nausea and vomiting in patients following laparoscopic surgery, on the other hand, had mixed findings. In light of these considerations, we decided to conduct a meta-analysis on the effectiveness of palonosetron throughout the postoperative recovery period. One of our key objectives is to determine if there are any statistically significant differences in the incidence of PONV (6, 24, and 48 hours after surgery) and the occurrence of adverse effects [10] at different time points after surgery

The article "Effect of Palonosetron on Physical Symptoms of Surgical Patients: A Systematic Review and Meta-Analysis" was published in 2022. Journal: Comput Math Methods Med.

## 2. Methods

### 2.1. Search Strategy

According to the Preferred Reporting Items for Systematic Reviews and Meta-Analyses (PRISMA) statement 5, this study satisfied all of the criteria for inclusion in a systematic review. For the terms “palonosetron,” “dexamethasone,” “surgery,” and “anesthesia,” we searched PubMed, the Cochrane Central Register of Controlled Trials (CENTRAL), EMBASE (Ovid), the Cumulative Index to Nursing and Allied Health Literature (CINAHL), Google Scholar, the Web of Science citation index, the US clinical trial register, the UK clinical trial register, the Australia and New Zealand clinical trial register, and the US clinical trial register. Additionally, we did not place any language limits on the literature search at the time of the investigation because we did not believe that they were required. All searches were carried out separately by two writers, and any inconsistencies that were detected after the search process had been completed were examined and rectified as appropriate.

### 2.2. Study Selection

It is included in this research because there are randomized control trials (RCTs) that included adult patients (16 years or older) who underwent surgery under general or neuraxial anesthesia. In this study, the intervention was the perioperative administration of palonosetron for the prevention of postoperative nausea and vomiting (PONV), while the control was the administration of other medications. It was found that the incidence of PONV and the requirement for rescue antiemetics within 24 hours were the most interesting. It was also found that the incidence of PONV within 6 hours and the incidence of PONV after 48 hours were both interesting.

### 2.3. Data Extraction

It was decided to use a standard proforma for the data extraction procedure, which was evaluated and confirmed by two authors independently over the course of the study. Additionally, the data extraction method covers the research design (such as the kind of surgery, the type of anesthetic, and the time and dose of palonosetron), as well as the study's findings (such as the author, year, and PubMed ID) (PONV, the need for rescue analgesia, and the results described in the research are all factors to consider). When outcome data was lacking, it was required to contact study authors via email in order to get more information; this was done many times in order to improve the number of replies obtained. For the purpose of analyzing clinical studies, we employed the RoB 2: Cochrane risk of bias assessment for randomized trials, which has been modified from its previous version, and it is now comprised of a 6-item questionnaire developed by the Cochrane Collaboration. There is a risk rating associated with each item. The risks are divided into three categories: low, moderate (some concerns), and high risk. At both the study and outcome levels, potential bias was examined, with all assessments carried out independently by two authors and any inconsistencies addressed and resolved with the assistance of a third author.

The article "Effect of Palonosetron on Physical Symptoms of Surgical Patients: A Systematic Review and Meta-Analysis" was published in 2022. Journal: Comput Math Methods Med.

### 2.4. Statistical Analysis

For any outcomes that were reported in more than one study, a meta-analysis was conducted to determine their significance. However, other than that, the findings were presented in a descriptive way. The Nordic Cochrane Centre and the Cochrane Collaboration used Review Manager (RevMan) version 5.3 for the pooled analysis, which was conducted by the Cochrane Collaboration (Copenhagen: Nordic Cochrane Centre and The Cochrane Collaboration, 2014). Resulting from the fact that the consequences are diametrically opposed, we used the Mantel-Haenszel approach to estimate our risk ratios (RRs). To assess the clinical importance of the data, we also counted the number of patients who would have required to be treated (NNT). The research was carried out in line with the random effect model. According to the sixth version of the Cochrane Handbook for Systematic Review of Interventions, the *I*^2^ statistic was employed to assess heterogeneity; a higher proportion indicates a greater degree of heterogeneity. It is probable that 0–40% of the variation is not significant, 30–60% represents moderate heterogeneity, 50–90% represents considerable heterogeneity, and 75–100% represents huge variability. As part of the sensitivity analysis, we deleted studies one by one and investigated whether or not the aggregate findings altered as a consequence. We discovered that they had no effect on the overall results. In addition, we performed a trial sequential analysis (TSA) of the included trials, with our key outcomes acting as the primary outcome variables for the analysis (24-hour risk of PONV). TSA Viewer version 0.9, which is freely available on the Internet, was utilized to perform the statistical analysis in this study.

## 3. Results

### 3.1. Description of the Studies That Were Included

The search was finished as of the most recent update on September 1, 2021. During the course of our research, we looked at a total of 1080 scholarly articles as well as abstracts from 18 conferences. In the end, we were able to discover a total of 10 papers for inclusion after conducting an extensive review of the data and eliminating duplicates (Figure 1) (Figure 2). According to the findings of the study, the great majority of patients had two or more Apfel risk factors, according to the findings, with the vast majority of those persons being female. In 10 studies, surgery was conducted under general anesthesia that was delivered by inhalational masks. The 10 clinical study studies included patients who had had high-risk surgeries for PONV, including laparoscopies, thyroidectomy, and bariatric surgery, among other treatments. Detailed information about the features of each of the studies that were considered for inclusion in this study is provided in this part of Table 1. An illustrative illustration of the results of the risk of bias assessment may be seen on the next paragraph. According to the findings, the absence of allocation concealment was the most significant source of bias, followed by the failure to register for the study prior to the study's start and the failure to report study participants' follow-up using the Consolidated Standards of Reporting Trials diagram, which were found to be the second and third most significant sources of bias, respectively.

The article "Effect of Palonosetron on Physical Symptoms of Surgical Patients: A Systematic Review and Meta-Analysis" was published in 2022. Journal: Comput Math Methods Med.

### 3.2. Incidence of PONV throughout 24-Hour

All the studies have explored the effect of palonosetron on PONV after 24 hours compared with other drugs (Figure 3). The difference was statistically significant 95% CL confidence range 0.03–0.06. According to the results of the sensitivity analysis, the outcome did not alter when each of the studies was excluded from the analysis. Because of the broad variety of patient and surgical risk factors observed in the studies included in this evaluation, the quality of the evidence is considered to be moderate. Additional to this, we conducted a subgroup analysis of palonosetron 8 mg in comparison to other drugs administered at lower or higher doses (4–5 mg or 10-12 mg) (Figure 4). There was no statistically significant difference between the effect ratios of the three subgroups (8 mg palonosetron, 95 percent confidence interval: 0.02–0.05; 4–5 mg palonosetron, 95 percent confidence interval: 0.03–0.07; 10–12 mg palonosetron, 95 percent confidence interval: 0.02–0.10).

### 3.3. Incidence of PONV throughout a 48-Hour Period

Over the course of a 48-hour period, there were 6 investigations that reported the total incidence rate (Figure 5). Because of the wide range of severity ratings for PONV, it was decided not to conduct a separate investigation of the occurrences of PONV in this study. It was shown that palonosetron had a favorable pooled risk ratio for 48-hour PONV incidence, but it was not statistically significant 95 percent confidence interval: 0.89–1.44, Egger's regression *p* = 4.94. Because of the wide range of results, the evidence is of mediocre quality. In the post hoc subgroup analysis by dexamethasone dosage, we discovered that there were two trials that employed 4 mg dexamethasone, and these studies were included in the final analysis (Figure 6). Pooled findings from the 8 mg dexamethasone subgroup in the combination therapy cohort indicated a trend toward significantly lower PONV risk (95 percent confidence interval: -0.99–0.06); however, the 4 mg dexamethasone subgroup demonstrated that there was no statistically significant difference between palonosetron alone and palonosetron combined treatment (95 percent confidence interval: 0.55–0.88).

The article "Effect of Palonosetron on Physical Symptoms of Surgical Patients: A Systematic Review and Meta-Analysis" was published in 2022. Journal: Comput Math Methods Med.

### 3.4. Incidence of PONV during 6-Hour Period

There were five studies that looked at the incidence of PONV in the first six hours following surgery and published their findings in the medical literature (Figure 7). Take a look at the pooled risk ratio for PONV occurrence during a 6-hour period, we can see that it is not statistically significant. We think the reason is that in the first six hours, the patient is in the awakening period, and his life activities are very different from those in normal times. According to the trim-and-fill model, there would be no missing research papers. According to the results of the sensitivity analysis, the outcome did not alter when each of the studies was excluded from the analysis. A post hoc sensitivity analysis was conducted after this.

### 3.5. Effects of Plasma Motilin Concentration Changes

Motilin is a linear polypeptide composed of 22 amino acids discovered in 1966. It is secreted by endocrine Mo cells and can be released periodically during the digestive period to promote gastrointestinal motility and stimulate the secretion of pepsin. It and PONV symptoms have a close relationship (Figure 8). From the results, we can see that palonosetron has a great influence on the concentration of plasma motilin.

### 3.6. Adverse Events

There was an increase in the frequency of adverse events in ten of the studies, with headache and dizziness being the most frequently reported symptoms. In any of the studies, there was no statistically significant difference between the groups, and this was true in all of them. It was highlighted that multiple trials had shown a tendency toward fewer adverse events in the palonosetron plus dexamethasone group as compared to the control group, which we found to be true in some cases. This was in accordance with our conclusions (Figure 9).

### 3.7. Risk of Bias across Studies

There was no problem bias recorded, as seen in the state funnel picture in Figure 10. Embraced studies are conducted in a methodical manner, implying no bias. The three studies are small and are distributed near the bottom of the picture (Figure 10).

The article "Effect of Palonosetron on Physical Symptoms of Surgical Patients: A Systematic Review and Meta-Analysis" was published in 2022. Journal: Comput Math Methods Med.

## 4. Discussion

Comparing other drugs to palonosetron, palonosetron is a new-generation 5-HT3 antagonist that has shown higher antiemetic efficiency (a second-generation 5-HT3 antagonist) [11]. It is anticipated that palonosetron's use in clinical practice will grow as a consequence of the availability of its generic formulation as well as the anticipated cost decrease. PONV consensus guidelines recommend that patients with any risk factors for the disease get wide multimodal prophylaxis, according to the most recent consensus guidelines published by Navari [12]. Among the most frequently prescribed combinations, the 5-HT3 antagonist with dexamethasone is by far the most frequently prescribed combination. To be fair, as the expert panel pointed out, not all combination medications have shown higher effectiveness when compared to their component therapies. Over the course of a 24-hour period, adding dexamethasone in palonosetron, according to the results of this systematic review and meta-analysis, significantly decreased the requirement for antiemetic medication [13]. This means that when combined with dexamethasone, palonosetron may be more effective than palonosetron alone in terms of preventing PONV infection. The trial sequence analysis, in addition, reveals that the present data is adequate to provide moderate support; nevertheless, further research is necessary to increase the quality of the available evidence [14].

Based on the research, it seems that a combined preventive medication for PONV is useful in minimizing the occurrence of this illness [15]. The probability of PONV in 6 hours, 24 hours, and 48 hours was statistically significant different, according to the findings of a literature search [16]. A subgroup analysis suggested that adding 8 mg dexamethasone to palonosetron after surgery may result in a decrease in 24-hour PONV incidence [17]; however, there were only a few clinical trials to confirm our findings [18]. Scholars discovered that the incidence of 2-hour PONV was decreased following combination treatment in several studies, but since the literature quality is exceedingly poor due to the likelihood of publication bias, these results have low reference value [19]. A recent meta-analysis, on the other hand, showed that the combination of other medicines plus dexamethasone considerably decreased the probability of 24-hour PONV [20]. This difference might be caused by a number of additional factors, including but not limited to: Because ondansetron has a relatively short half-life (4 hours), it is expected that it will be more effective when combined with longer-acting antiemetics (such as dexamethasone) than when taken alone (whose half-life ranges from 36 to 54 hours). When compared to the medicine ondansetron, palonosetron is far more effective and has a longer half-life of more than 30 hours, making it a better therapeutic option. In this case, the use of dexamethasone is likely to expand the patient's margin of benefit.

The article "Effect of Palonosetron on Physical Symptoms of Surgical Patients: A Systematic Review and Meta-Analysis" was published in 2022. Journal: Comput Math Methods Med.

When it comes to severe nausea and vomiting, scuenti-emetic is frequently saved for the worst cases, although reported PONV may be mild and not need the use of antiemetic medicine [21]. If this is true, it suggests that a combination prophylactic may be more effective in avoiding nausea and vomiting that varies in intensity from mild to severe. Some previous study found that palonosetron and dexamethasone combine therapy reduces the risk of PONV. When the cumulative *Z* score was examined for the 24-hour PONV risk, it was discovered that it did not exceed the observation boundaries, as had been recommended by the research [22]. The findings of this study demonstrate that the present sample size is insufficient for the credible clinical evidence, and that further research may have an impact on the conclusions of this meta-analysis if the sample size is increased in the future. Despite the fact that this meta-analysis offers a number of significant benefits, it also have a number of significant drawbacks [23].

First and foremost, there is a great deal of variation between surgical method PONV risk, both of which are significant [24]. However, owing to the study number limitation, it is not feasible to completely address the heterogeneity using subgroup analysis due to the low number of studies available, making it impossible to fully address the heterogeneity using subgroup analysis. As a second point, owing to the limited amount of data currently available, it is not feasible to correctly differentiate between nausea and vomiting in the great majority of cases. This is due to a lack of sufficient data in the current data scarcity [25]. Most likely, this is the reason of the discrepancy between the findings about the threat of PONV and the necessity for rescue analgesia in this particular instance. For the last point, since most existing research has been conducted on female patients requiring intermediate to major surgery, it is likely that the results here will not apply to lower-risk day case surgical procedures that are performed on a more regular basis [26].

The fact that palonosetron prophylaxis is related with a considerable decrease in the requirement for rescue antiemetics in patients undergoing intermediate to high-risk surgery for PONV continues to be debated in the medical community [27, 28], the study found that it had only a small impact on the overall incidence of PONV in patients. According to the findings of the trial sequence analysis, more study on this topic is required in order to create more reliable clinical data.

The article "Effect of Palonosetron on Physical Symptoms of Surgical Patients: A Systematic Review and Meta-Analysis" was published in 2022. Journal: Comput Math Methods Med.

## Figures and Tables

**Figure 1:** Process of literature screening.

**Figure 2:** Summary of the results of the risk of bias.

**Figure 3:** Effect of palonosetron on PONV after 24 hours.

**Figure 4:** Different doses of palonosetron RIDIT.

**Figure 5:** Incidence rate of PONV after 48 hours.

**Figure 6:** Comparison of PONV risk of dexamethasone combination.

**Figure 7:** Comparison of 6-hour PONV.

**Figure 8:** Effect of palonosetron concentration on plasma motilin.

**Figure 9:** Comparison of adverse reactions.

**Figure 10:** Risk of bias assessment.

**Table 1:** Summary of 10 studies: author (years) participant surgery/anesthesia outcome.

Author (years)	Participants	Surgery/anesthesia	Outcomes
Adis (2009)	70 patients with cancer	Laparoscopic cholecystectomy under isoflurane/nitrous oxide GA	Headache and constipation were among the most commonly reported adverse events with the use of palonosetron
Ahn et al. (2016)	695 patients were included in the final analysis	Laparoscopic abdominal and pelvic surgeries under sevoflurane GA	Palonosetron was more effective than ramosetron, when the administration time for the 5-HT3 receptor antagonist was during the early phase of the operation
Srivastava et al. (2020)	64 patients, scheduled for middle ear surgery, were randomized into two groups	Laparoscopic cholecystectomy under sevoflurane GA	The combination of palonosetron-dexamethasone is superior to ondansetron-dexamethasone for the prevention of postoperative nausea and vomiting after middle ear surgeries
Fonseca et al. (2020)	60 individuals who underwent video cholecystectomy were randomized into three groups	Sevoflurane þ remifentanil	The present study showed evidence that palonosetron is superior to the drugs compared regarding a protracted antiemetic effect and less requirement of rescue drugs, mainly related to its ability to completely inhibit the uncomfortable symptom of nausea
Liu et al. (2018)	129 patients were included in the final analysis	Laparoscopic cholecystectomy under isoflurane/nitrous oxide GA	Palonosetron is not more efficacious than ondansetron in the prevention of early PONV. However, palonosetron was more efficacious than ondansetron in the prevention of vomiting after laparoscopic surgery
Lee et al. (2019)	51 adult patients	Bariatric surgery under sevoflurane GA	LBW-based dosing might be suitable for high-weight patients to avoid possible underdosing. Nevertheless, the current fixed dosing of palonosetron is acceptable for adult patients with normal weight
Grigio et al. (2020)	100 patients according to a random number generator	Laparoscopic cholecystectomy under isoflurane/nitrous oxide GA	The addition of aprepitant as a third antiemetic resulted in no significant reduction in the incidence of PONV in this population. However, the incidence of PONV was reduced in relation to the general population
Gouveia et al. (2020)	Involving 80 female patients	Thyroid surgery under sevoflurane/nitrous oxide GA	A body weight-adjusted dose of palonosetron was as effective as 75 *μ*g for preventing PONV for 48 h in obese female patients who underwent breast surgery. Hence, the fixed dose may be preferable to the body weight-adjusted dose
Song et al. (2017)	146 patients were randomly allocated	Laparoscopic abdominal or pelvic surgery under sevoflurane GA	Compared with palonosetron, ramosetron may be superior for reducing PONV severity, especially in patients with ABCB1 3435TT or 2677TT genotype
Kang et al. (2018)	274 adults	Laparoscopic surgeries under sevoflurane GA	The combined use of prophylactic palonosetron before anesthetic induction and sugammadex as a reversal of neuromuscular blockade are associated with a reduction in the incidence of PONV in patients undergoing MVD under propofol-maintained anesthesia

The article "Effect of Palonosetron on Physical Symptoms of Surgical Patients: A Systematic Review and Meta-Analysis" was published in 2022. Journal: Comput Math Methods Med.

## Data Availability

The datasets generated during and/or analyzed during the current study are available from the corresponding author on reasonable request.
